The article "Alpha-Bulges in G Protein-Coupled Receptors" was published in 2014. Journal: Int J Mol Sci.

# Alpha-Bulges in G Protein-Coupled Receptors

**DOI:** 10.3390/ijms15057841

**Published:** 2014-05-06

**Authors:** Rob van der Kant, Gert Vriend

**Affiliations:** Centre for Molecular and Biomolecular Informatics, Radboud University Medical Centre, Geert Grooteplein 26-28, 6525 GA Nijmegen, The Netherlands

**Keywords:** GPCR, π-helix, α-bulge, GPCR activation, random forest, structure-function

## Abstract

Agonist binding is related to a series of motions in G protein-coupled receptors (GPCRs) that result in the separation of transmembrane helices III and VI at their cytosolic ends and subsequent G protein binding. A large number of smaller motions also seem to be associated with activation. Most helices in GPCRs are highly irregular and often contain kinks, with extensive literature already available about the role of prolines in kink formation and the precise function of these kinks. GPCR transmembrane helices also contain many α-bulges. In this article we aim to draw attention to the role of these α-bulges in ligand and G-protein binding, as well as their role in several aspects of the mobility associated with GPCR activation. This mobility includes regularization and translation of helix III in the extracellular direction, a rotation of the entire helix VI, an inward movement of the helices near the extracellular side, and a concerted motion of the cytosolic ends of the helices that makes their orientation appear more circular and that opens up space for the G protein to bind. In several cases, α-bulges either appear or disappear as part of the activation process.

## 1. Introduction

G protein-coupled receptors (GPCRs) are important targets for the pharmaceutical industry and have consequently been studied extensively *in vivo*, *in vitro*, and *in silico*. Their importance is illustrated by the fact that PubMed [1] lists around 500 reviews relating to GPCRs every year. The first three-dimensional structure of a GPCR was solved in 2000 [2], and recent years have seen a flurry of GPCR structures [3] being solved, published and deposited in the PDB (Protein Data Bank) [4]. Nearly all the GPCR structures solved so far are from the rhodopsin-like family—normally referred to as the Class A GPCR family. This article exclusively examines Class A GPCRs, so each time the acronym GPCR is used, it should be interpreted as “Class A GPCR”.

GPCRs possess seven transmembrane helices that traverse the membrane as illustrated in Figure 1. The *N*-terminus is located extracellularly and the *C*-terminus is located in the cytosol. Each helix contains at least one highly conserved residue (see Figure 1). These conserved residues are commonly used to anchor GPCR sequence alignments using the soon to be abandoned concept that “there are no insertions and deletions in helices” [5,6].

The article "Alpha-Bulges in G Protein-Coupled Receptors" was published in 2014. Journal: Int J Mol Sci.

In the year 2000, the first structure of a GPCR was solved experimentally [2]. This structure not only revealed a series of surprises but also confirmed [8] or falsified [9] a series of previous hypotheses. Other hypotheses [10] were proven right in concept but wrong in detail. After the second GPCR structure had been solved (the β2 adrenergic receptor [11]), the floodgates opened, with the result that over the last few years we have on average been able to study one new GPCR structure every few months. The most frequent source of newly solved GPCRs has been the Stevens Lab [3].

GPCRs are notoriously difficult to crystallize. They are membrane proteins and therefore have large hydrophobic surfaces that are prone to nonspecific binding. However, it is perhaps even more important to realize that most GPCRs exhibit constitutive activity, which means they are highly mobile, continuously moving in and out of the active state. Consequently, GPCR crystallographers not only need to cope with the classical membrane crystallization problem of sticky hydrophobic surfaces, they also need to fixate the GPCR in one of its many marginally stable conformations. The sticky surface problem is frequently addressed by adding amphiphiles, while increasing the hydrophilic surface is often done by cloning lysozyme covalently into the GPCR. This covalent cloning is typically done between helices V and VI (e.g., as in the β2 adrenoceptor [11]), but lysozyme has also been cloned-in at other locations (e.g., the β2 adrenoceptor in which lysozyme has been fused to the *N*-terminus [12]). Other molecules are also being used for this purpose [13]. The GPCR mobility issue has been reduced by adding strong binding ligands (e.g., PDBid = 3eml [14]), nanobodies (e.g., PDBid = 3p0g [15]), G proteins (e.g., PDBid = 3sn6 [11]), and by mutating the residues that are most involved in the activation process—for example, the β1 adrenoceptor (PDBid = 2vt4 [16]) or the adenosine A2A receptor (PDBid = 3rey [17]). All these modifications have an influence on the structure. Figure 2 shows a series of examples of non-native interactions observed in GPCR structures. An associated web page [18] holds pictures of the 84 GPCR structures presently available with the modifications and non-native interactions indicated.

When a GPCR structure deviates from the canonical situation shown in Figure 1, it is important to consider whether the deviation is an interesting finding or a crystallization artifact. For example, in the recently solved structure of the NTS1 neurotensin receptor (PDBid = 4grv [19]) we observed that helix VIII is barely present and what can be seen of it appears to be displaced. This could be an interesting finding, but it seems more likely that a large number of crystal packing contacts (see Figure 3) has caused helix I to occupy the canonical space of helix VIII, causing helix VIII to find another stable position packing against the cloned-in lysozyme structure [19].

The article "Alpha-Bulges in G Protein-Coupled Receptors" was published in 2014. Journal: Int J Mol Sci.

Mason *et al.* [20] found that upon receptor activation, the volume of the ligand binding site decreased by ~40 Å^3^ for the β1 and β2 adrenoceptors and by ~90 Å^3^ for the purinergic A2A receptor. This indicates that agonists stabilize a receptor conformation in which the extracellular sides of certain helices are closer together. This finding, combined with the finding of the “see-saw” like motions of helices [21,22], results in a model that can be compared to the mechanism of a clothespin. This model is explained in Figure 4.

GPCR structures have been modified in many different ways to aid crystallization, but fortunately, because many different crystallization methods have been used, we can still extract an overall picture by observing trends in large numbers of GPCR structures. After dealing with sequence insertions and deletions caused by α-bulges and short stretches of π-helix and 3_10_-helix, we can unambiguously assign 203 residues that are common to all GPCR structures, all of which we can be reasonably sure are homologous. We have measured the 20,503 pair-wise distances between these 203 residues in 69 GPCR structures, and we have analyzed these distances using the random forest (RF) method. One of the scientific possibilities offered by the RF method when applied to a very large set of observations is detection of those observations that are most supportive for a hypothesized classification. We produced a series of structure classifications, each consisting of either two or three groups. Examples are: dark-state rhodopsins versus other receptors in the inactive state; receptors with a G protein or nanobody bound at the cytosolic side versus all others; and adenosine receptors with bound inverse agonists, antagonists or agonists.

The results shed new light on the GPCR activation process, on the roles of many individual residues, and on the helix motions. They also shed new light on α-bulges and their role in the dynamic processes related to GPCR activation. Upon activation (either by G-protein binding or by other means) helices III and VI separate at the cytosolic side, while helix III translates slightly in the extracellular direction [18].

Helical distortions play a major role in the overall fold of GPCRs. Most GPCRs possess α-bulges [24–30] in helices II and V, but they are also observable in most other helices in one or more GPCRs; only in the lipid receptor structures did we not detect any α-bulges. The highly conserved α-bulges often mentioned in helices II and V are not present in all GPCR structures, and when they are present, their locations are not always strictly conserved. In the second transmembrane segment (TM2), for example, the proline pattern is not conserved in sequence space. When present, it may be located at position 232, 233, or 234. In 2009 Devillé *et al.* [29] proposed that an indel led to two structural motifs for helix 2: bulged receptors with a proline at position 233 or 234 or a kink in receptors with a proline at position 232. In the structures available today, though, the proline in TM2 is structurally conserved and the observed sequence variability is caused by the absence or presence of an α-bulge. This sequence motif is particularly important for predicting the presence of bulges near the ligand-binding site, which in turn is crucial for homology modeling. Figure 5 shows how in the trace amine subfamily in the GPCRDB [5] a bulge is observed near position 229 in about half of all family members.

α-Bulges tend to remain stable in molecular dynamics simulations, indicating that these bulges represent (at least) a local energy minimum (DE Gloriam, personal communication).

The article "Alpha-Bulges in G Protein-Coupled Receptors" was published in 2014. Journal: Int J Mol Sci.

We will argue that the role of prolines near the kinks in the helices is different to that previously thought. Overall, our results lead to a series of new hypotheses that are amenable to experimental validation.

## 2. Results

The way we use the RF method to analyze GPCR structure characteristics in distance space requires that the hypotheses put forward logically lead to classifications of existing GPCR structures involving a limited number of groups. Any hypothesis related to the activation process will be a good candidate, because the GPCR structure community has been working hard to shed light on this process by solving the structures of GPCRs with bound agonists, partial agonists, *etc.* and GPCR structures in the presence and absence of G proteins.

Visual inspection reveals that residue Tyr733 is displaced the most between active and inactive structures, with widening of the gap between helices III and VI also being closely associated with activation. In total, 202 distance vectors relate to displacement of the Tyr733 residue. However, almost eight times this number of vectors contribute to the relative displacement of helices III and VI. This asymmetry between the number of distance vectors related to displacement of Tyr733 and the number of distance vectors related to displacement of helices III and VI causes artifacts in the RF computations [32,33]. We therefore iteratively searched for the pair of distance vectors that had the highest Pearson correlation coefficient, randomly removing one of the two vectors during each iteration. This process was repeated until no two distance vectors had a Pearson correlation coefficient higher than 0.90, resulting in removal of around 80% of the vectors. The RF determination of the distance vectors most representative for the differences between active and inactive structures are projected on 1F88 in Figure 6. The yellow lines in Figure 6 represent distances that are shorter in the active state GPCRs than in the inactive ones. Most of the yellow vectors in Figure 6 are caused by a small but systematic displacement of helix III towards the extracellular side in the active state structures. The magenta lines represent distances that increase upon activation. These mainly involve the cytosolic side of helix VI, which undergoes an outward motion away from the rest of the helix bundle upon activation.

The article "Alpha-Bulges in G Protein-Coupled Receptors" was published in 2014. Journal: Int J Mol Sci.

Tyr733, which is located at the intracellular side of helix VII, is the most important single residue to classify receptors as either being in the active state or the inactive state. It has been hypothesized [2,8,34–36] that this highly conserved residue stabilizes the active state by stabilizing the open conformation of the “ionic lock” formed by Arg340 and Glu600. During activation, the local backbone around Tyr733 undergoes a complicated reorganization, part of which involves the appearance/disappearance of an α-bulge.

When we use RF to determine the most significant distance differences between active and inactive GPCR structures, we find that many of these involve a residue in helix III. Visual inspection of superposed structures in the active and inactive state reveals that helix III is slightly displaced towards the extracellular direction in the activated GPCRs. Helix III is also slightly more wound up in the activated state. We also observe a correlation between truncation of the *N*-terminus and an outward movement of the extracellular side of helix I, as illustrated in Figure 7.

Although many articles have been published about the role of prolines in inducing kinks in helices (e.g., [37–43]), we do not believe that prolines actively induce these kinks. We believe that they merely allow for them. Nevertheless, the suggestion that a relationship exists between prolines, kinks, and the mobility that is necessary for GPCR activation continues to be a prominent part of experimental studies. However, our structural comparisons between GPCRs in the active and inactive form do not fully support this suggestion, as is illustrated in Figure 8, in which the active form of the β2-adrenoceptor is superposed on its inactive form. Figure 8 illustrates that the structural differences observed in the helices are not related one-to-one to the presence of prolines. The major hinge point is located near the kink in helix VI, but this helix does not bend in the middle; it undergoes a full-helix rotation. The blue and red helix VI in Figure 8 can be superposed on all 28 Cα atoms (including the residues in the irregular area near the ligand binding site) with an RMS displacement of only 0.9 Å.

The article "Alpha-Bulges in G Protein-Coupled Receptors" was published in 2014. Journal: Int J Mol Sci.

In every kinked helix, a highly conserved proline is found near the kink. Whenever there is a non-helical element in the middle of a helix, a proline starts the “rest” of that helix. These non-helical elements can take the form of an α-bulge or a short 3_10_ helix. Our supposition is that prolines do not induce kinks, as has often been suggested, but merely facilitate the non-helical element in the middle of the helix and ensure that the transmembrane domain can, after the irregularity, continue as a normal α-helix. In Figure 8 we see that for all cases the irregularities are highly similar in the active and inactive form, except for helix VII. In the inactive state this helix has a large stretch of residues forming a highly irregular helix, whereas in the active state the helix is more regular. The fact that helix VI rotates in its entirety rather than bending at the kink near the proline further adds to the idea that the relationship between prolines and kinks is not as simple and direct as has often been suggested.

Table 1 lists the α-bulges observed in the seven transmembrane helices in the 84 GPCRs studied. Figure 9 shows the distribution of secondary structure types over all the residues that these 69 structures have in common. The often mentioned [24–30] α-bulges in helices II and V are present in nearly all GPCRs, but they are not as highly conserved as some other features, and their locations are not conserved. Especially in helix V, many more irregularities are observed—and the S1P-lipid receptors lack the α-bulge in helix V. Interestingly, this receptor does not have the otherwise conserved proline at position 520. This finding might even indicate an alternative way for the lipid ligand to enter the active site, because the flexible ligand can perhaps enter directly from the membrane between helices IV and V [18]. Figure 10 illustrates the variability of the bulges observed in helix V.

Most structures have an α-bulge in the middle of helix II, notable exceptions being opioid, CXCR4, CCR5, and lipid receptors. Visual inspection of structures containing the bulge in helix II does not suggest a functional role for it despite that it is located at the same depth in the membrane as the ligand binding site. Squid rhodopsin (PDBid = 2z73 [47]) has an α-bulge at the extracellular side of helix II that is absent in bovine rhodopsin.

The article "Alpha-Bulges in G Protein-Coupled Receptors" was published in 2014. Journal: Int J Mol Sci.

The α-bulge after Tyr733 is present in all GPCR structures except the β1 and β2 adrenoceptors. The absence of this bulge in β1 and β2 adrenoceptors is correlated with the presence of a proline at location 808 (in the corner between helices VII and VIII). It therefore appears that both the bulge and the proline can facilitate a similar displacement of Tyr733. Figure 11 illustrates these effects. This bulge may be “needed” to allow tyrosine 733 to bend inwards and assist in stabilization of G protein binding to the GPCR. The word “needed” should be read with caution, as there is no indication of a causal relationship between the two observations.

Figure 12 shows the bulges in helix IV in the CXCR4 chemokine receptor (PDBid = 3odu [48]) and the M2 muscarinic acetylcholine receptor (PDBid = 3uon [49]). At present, it is not possible to evidentially associate these bulges with any particular function, although it could be speculated that they play a role in dimer formation.

For the adenosine 2A receptor, structures are available bound to inverse agonists, antagonists, and agonists. Unfortunately, no structure is available yet for this receptor with a bound G protein. Figure 13 shows the superposition of the ten available structures for the adenosine 2A receptor and indicates that in most cases the differences between structures with a bound inverse agonist and structures with a bound antagonist are small. However, the structural differences are larger when either of these two groups is compared to structures with a bound agonist. Most of these structural differences seem to agree with the clothespin mechanism [53] but the displacements seen for the cytosolic side of helix V are surprising. When going from a bound inverse agonist to an antagonist we observe an inward motion of helix V, and upon binding of the agonist we observe an outward motion. We have no explanation yet for this counter-intuitive phenomenon.

Figure 13 shows differences in the helices observed in globally superposed structures. Figure 13 shows the same helices in the same colors with the helices superposed locally. This local superposition reveals that helix VI rotates as a whole rather than its cytosolic side bending outwards (see Figure 14). Helix III becomes more regular and less bent upon binding an agonist. Helix V winds up more tightly going from the inverse agonist, via the antagonist, to the agonist bound structures.

The article "Alpha-Bulges in G Protein-Coupled Receptors" was published in 2014. Journal: Int J Mol Sci.

Many structures are available for the β2 adrenoceptor family, including structures with bound agonists, antagonists, and inverse agonists. We also have a structure for a bound G protein trimer, and a structure with a nanobody bound in such a way that similar displacements are observed. This diversity of β2 adrenoceptor structures allows an in-depth study of how they move during different phases of the activation process. Figure 15 shows differences in the helices observed in globally superposed structures.

## 3. Discussion

Over one hundred GPCR structures are available in the PDB. These structures relate to more than ten different GPCRs that have been solved with and without nanobodies or G proteins bound to them; with different ligands bound to them, and with different modifications to achieve crystallization. All these structures contain at least some artifacts due to crystallization. Binding a ligand or a G protein leads to structural changes such as helix displacements or rotamer flips in residues, but it is sometimes hard to separate these endogenous activation-related structure changes from those caused by crystallization artifacts. We used the variable importance score of the Random Forest (RF) method to elucidate which distances differ systematically as a function of motions associated with different phases of the GPCR activation process. However, the results of this approach cannot be taken at face-value, because we manually defined which structures were in the active or inactive state (G protein bound, or nanobody bound at the same location) and then used the RF method to determine which interatomic distances differ most systematically between the defined states. Similarly, a comparison of structures with bound agonists, antagonists, or inverse agonists is only as good as the determination of whether the bound compounds indeed are an agonist, *etc.* In addition, there is the risk that we may have missed a confounding variable—for example, the possibility that inverse agonists only bind to structures in which a certain mutation has been introduced.

The comparison between active structures and inactive structures, and between structures with an agonist bound and structures with an inverse agonist bound, revealed several interesting systematic movements. The strongest systematically observed effect in GPCR activation is an inward motion of Tyr733. It has been hypothesized [2,8,34–36] that this residue stabilizes the active conformation by interacting with Arg340, thereby stabilizing the open conformation of the “ionic lock” comprising Arg340 and Glu600. The outward motion of the intracellular side of helix VI is also systematically related to stages of the activation process, and is more a rotation of the entire helix then it is a bending of the helix at the kink near W618 and P620.

The article "Alpha-Bulges in G Protein-Coupled Receptors" was published in 2014. Journal: Int J Mol Sci.

Compared to structures in the inactive state, structures in the active state show an upward (towards the outside of the cell) displacement of helix III combined with a hard to describe screw motion that makes the extracellular part of helix III a more regular α-helix. The extent of this upward displacement differs from case to case.

Agonist binding brings helices V–VII closer to each other around the ligand-binding site. Activation and G-protein binding are associated with a displacement of the intracellular part of helix VI that creates the crevice in which the G protein binds. Helix VI, however, does not have a hinge-point where the bending angle of the helix changes. The helix itself stays rigid but it rotates in such a way that its cytosolic side moves outwards. Combined with the regularization of helix III, and the known constitutive activity of many GPCRs in the absence of agonists, we see similarity to a clothespin in the model for G protein activation. GPCRs are mostly in the inactive conformation (clothespin closed) and occasionally in the active conformation (clothespin open), in which state they can activate a G protein (catch the laundry). Agonist binding and G protein binding both stabilize the active conformation. The activating ligand keeps the extracellular sides of helices V–VII close together and straightens helix III, while also moving helix III upwards, towards the extracellular side. The other helices do not bend at their hinge points but maintain their same general local orientation. It could be hypothesized that the upward movement of helix III makes it easier to break the ionic lock. During GPCR activation, Arg340 flips upwards, where it is maintained in position by interactions with Tyr733 and Tyr528. This creates a crevice at the intracellular side of the receptor in which the *C*-terminal end of a G protein’s α-subunit can dock. After binding to the activated GPCR, the G protein exchanges its bound GDP for a GTP and activates downstream pathways. An inverse agonist keeps the GPCR in its inactive state by pushing the extracellular sides of the helices outward, thus keeping the cytosolic sides of the helices close to one another.

## 4. Methods

GPCR structures were extracted from the PDB [58] and stripped of water, crystallization additives, multimeric partners, G proteins, cloned-in lysozymes, antibodies, *etc.* They were renumbered using the GPCRDB numbering scheme [59] which has the advantage of allocating identical residue numbers to homologous residues, making it easier for many computer programs to deal with them. For example, the Utopia-GPCRDB intelligent PDF-reader [60] directly couples GPCR-related articles to the GPCRDB [61] information system, making it very easy to place information extracted from an article in the wider context of GPCR knowledge. For example, this article can be read most productively using the Utopia-GPCRDB intelligent PDF-reader, which can be downloaded from the GPCRDB [61].

The article "Alpha-Bulges in G Protein-Coupled Receptors" was published in 2014. Journal: Int J Mol Sci.

Unless mentioned otherwise, global structure superpositions were performed using the YASARA (YASARA Biosciences, Vienna, Austria) [44] implementation of the Mustang structure alignment program [62]. Local superpositions were produced with the WHAT IF [63] superposition module [64] that is integrated into YASARA. The superposition of single helices using only Cα atoms of corresponding residues (thus neglecting bulge residues when one superposition partner does not possess that bulge) was performed using a variant of the WHAT IF superposition module specifically adapted for the purpose.

Analyses were performed using the randomForest module [65] in the R [66] package. Variable importances for predefined classes were determined using standard parameters and ntree = 1000, importance = TRUE. Variables were sorted with the *G*_ini_ importance parameter as sorting key.

α-Bulges were detected with a rewritten version of DSSP [67]. This rewritten version, DSSP 2.0, produces >>99.9% the same results as the now thirty-year old original DSSP 1.0 program written by Kabsch and Sander when α-bulges (also often called π-helices [26]) are not counted. Table 1 lists the structures used and their α-bulges.

DSSP 2.0 is freely available through the Centre for Molecular Bacteriology and Infection (CMBI) structure facilities [68] web pages [69] or directly from the DSSP FTP site at [70]. All structures mentioned in this study, and an extensive study of the effects of mutations and crystallization additives on the structures, are available at [18]. This website also holds many methodological details that are beyond the scope of this article.

## 5. Conclusions

We have shown that α-bulges are a prominent feature of GPCRs and that the bulges in helices II and V are highly conserved, albeit varying in type, and in helix V also varying in location. We also observed bulges in helices IV and VII. In several cases, the presence or absence of these bulges is directly linked to the activation process, but in other cases this conclusion awaits experimental validation. Although α-bulges have so far largely eluded the interest of the GPCR research community, we hope that this short summary of our observations will stimulate experiments aimed at shedding light on their precise functional role.

The article "Alpha-Bulges in G Protein-Coupled Receptors" was published in 2014. Journal: Int J Mol Sci.

## Figures and Tables

**Figure 1.** Overview of G protein-coupled receptors (GPCR) helix bundle with conserved residues indicated. In most GPCR sequences, we find the following conserved residues (first digit indicates the helix number; see the GPCRDB [5,6] or other GPCR systems like the Glycoprotein-hormone Receptor Information System (GRIS) [7] for a detailed discussion of the numbering system): Gly129, Asn130, Leu220, Asp224, Asn729, Pro730 (in the ion pocket that is involved in signalling between the ligand binding site and the G-protein binding site); Cys315 (which forms a Cys–Cys bridge with Cys446 in the loop between helices IV and V), Asp339, Arg340, Tyr341 (the DRY motif, involved in activation), and Tyr528 (involved in G protein interactions); Trp 420 (purple, just visible behind the ion pocket residues; likely involved in cholesterol binding, perhaps involved in dimer contacts), Pro520, Cys617, Trp618, Pro620 (involved in ligand interaction and trigger and/or hinge for motions needed for activation) Tyr733 (just underneath the ion pocket, swings from proximity of ion pocket into direction of DRY upon activation). Rhodopsin (PDBid = 1f88 [2]) has been used for this figure.

**Figure 2.** Examples of crystallization artifacts. (**A**) The turkey β1-adrenoceptor, PDBid = 2vt4 [16]. The asymmetric unit contains a dimer of non-natural up-side-down dimers. The A subunit in the first dimer is shown in blue while the other three monomers are shown in purple. Crystallization additives are shown in a ball representation. Residues in other molecules in the crystal that have at least one atom within 10 Å from any of the four subunits in the asymmetric unit are shown as a purple stick model; (**B**) Ribbon representation of bovine rhodopsin, PDBid = 1f88 [2]. All residue positions mutated for thermostabilization in any of the structures mentioned in this article are shown in a red ball-representation; and (**C**) Trace representation of the β2 adrenoceptor, PDBid = 2r4s [23] shown in dark blue bound to an antibody shown in magenta. The β2 adrenoceptor with PDBid = 3ny9 [12] that does not bind anything in this region is superposed and shown in light blue. Both are bound to inverse agonists. The antibody distorts helix VIII resulting in a bulge in 2r4s (shown in red) followed by an anti-bulge (3_10_ helix) at the location where 3ny9 has a normal helix (shown in green).

**Figure 3.** The structures of the neurotensin 1 (NTS1) receptor (red; PDBid = 4grv [19]) and rhodopsin (blue; PDBid = 1f88 [2]). The lysozyme that is cloned between helices V and VI in NTS1 is partly shown (in yellow). Helix VIII is shown in dark blue in rhodopsin and in green in NTS1. The purple lines indicate crystal packing contacts made by helix I in NTS1.

The article "Alpha-Bulges in G Protein-Coupled Receptors" was published in 2014. Journal: Int J Mol Sci.

**Figure 4.** Mechanism of GPCR activation. Agonist binding (**1**) induces inward motions (**2**) of the extracellular side of helices V–VII. This is accompanied by an outward movement of the cytosolic side of helices V–VII (**3**), allowing the G protein (shown as solid blue blob) to bind (**4**) and become activated (**5**). Obviously, there is no fixed order in the motions. The determination of what moves where depends largely on the superposition method used.

**Figure 5.** Fourteen consecutive residues in helix II (starting at the conserved L at position 220) extracted from the trace amine sequence alignment from the GPCRDB. From left to right the columns contain the GPCRDB sequence number, the consensus sequence at that position, and the amino acid at that position in each of the 61 sequences in the GPCRDB trace amine family 16. Figure copied with permission from Isberg *et al.* [31].

**Figure 6.** Distances found to be important by the random forest method to separate active from inactive structures mapped on rhodopsin (PDBid = 1f88 [2]) looked at from the intracellular side. The distances indicated in magenta increase upon activation; distances indicated in yellow decrease upon activation.

**Figure 7.** Helix I extracted from a structural alignment of 69 structures in YASARA’s [44] Cα trace representation. The structures from which the *N*-terminal domain was removed (and sometimes also a small part of the extracellular end of this helix truncated), display an outward displacement of helix I away from the transmembrane helix bundle.

**Figure 8.** β-2 adrenoceptor in the active state (PDBid = 3sn6 [11]; red) superposed on the inactive state (PDBid = 3ny8 [12]; cyan). The superposition was performed with the WHAT IF superposition module and involved 239 residues that matched with an RMS Cα displacement of 1.34 Å. Ligands, sugars, G proteins, *etc.* are not shown for clarity. Prolines are colored green. The major differences observed are in helices V and VI in the lower left of the figure. In the active form, helix V is much longer and the cytosolic half of helix VI is rotated outwards by about 30 degrees (please note that this involves a rotation of the entire helix, not just the cytosolic half). Further large differences are seen in helix VII (in the centre) and in the corner between helices VII and VIII. The different orientation of helix I (right most helix) in the two structures is most likely caused by crystal packing artifacts.

**Figure 9.** Secondary structure distribution for residues that are common to the 69 structures used in this study. Blue: α-helix; yellow: α-bulge/π-helix; purple: 3_10_ helix; orange: loop, strand, and turn. Each vertical bar is 69 residues high and the fraction of the bar in a certain color corresponds to the fraction of residues with the corresponding secondary structure. Secondary structures were determined with DSSP 2.0. The plot contains all transmembrane residues plus a few residues into the loop areas that all 69 structures have in common. In most α-bulge areas, one residue is therefore not counted. Small white bars represent the elements between the transmembrane regions that are not structurally conserved throughout the 69 structures. The central part of helix VII is either a regular helix, or consists of a stretch of 3_10_ helix combined with a bulge or similar irregularity. Despite bulges and 3_10_ stretches, the part of helix VII that ends with the conserved NP motif at positions 729 and 730 always has equally many residues so that no residue numbering differences can be observed between receptors.

The article "Alpha-Bulges in G Protein-Coupled Receptors" was published in 2014. Journal: Int J Mol Sci.

**Figure 10.** The area around the bulge in helix-V. The S1P lipid receptor (orange, PDBid = 3v2y [45]) does not have α-bulges in helix V and is given as a reference. Rhodopsin (magenta, PDBid = 1f88 [2]) and the adenosine-2A receptor (blue, PDBid = 3eml [46]) have an α-bulge (A) between positions 516 and 517; and the adenosine-2A receptor has an extra bulge (B) between positions 511 and 512. Side chains of residues at position 520 are shown. Rhodopsin and the adenosine-2A receptor have a proline at position 520. The S1P lipid receptor, which does not have bulges in helix V, does not have a proline at position 520. Time will tell if this correlation is accidental or causal.

**Figure 11.** Structural variability in the intracellular part of helix VII near residue Tyr733. In all four panels the cytosolic side of helix VII and the beginning of helix VIII are shown as a trace model and the Tyr733 side chain is shown as a stick model. In all four panels helix VIII points to the right. (**A**) Cyan represents inactive rhodopsin (PDBid = 1f88 [2]), blue represents inactive β2 adrenoceptor (PDBid = 3ny9 [12]). After Tyr733, rhodopsin forms a normal helix and the β2 adrenoceptor forms a 3_10_ helix, which is followed by a proline at the beginning of helix VIII. In the Panels **B**–**D**, cyan represents the inactive state, red represents the active state; (**B**) Adenosine A2A receptor. Cyan: PDBid = 3eml [46]. Red: PDBid = 2ydo [14]; (**C**) β2 adrenoceptor. Cyan: PDBid = 3ny9 [12]. Red: PDBid = 3sn6 [11]; and (**D**) Rhodopsin. Cyan: PDBid = 1f88 [2]. Red: PDBid = 3cap [50]. In rhodopsin and the adenosine A2A receptor, a bulge is formed upon activation. In the β2 adrenoceptor the inactive state has a 3_10_ helix, which becomes a normal helix upon activation.

The article "Alpha-Bulges in G Protein-Coupled Receptors" was published in 2014. Journal: Int J Mol Sci.

**Figure 12.** Bulges in helix IV. **Left**: CXCR4 chemokine receptor (blue; PDBid = 3odu [48]) superposed on the delta opioid receptor (cyan; PDBid = 4ej4 [51]) as reference. The CXCR4 chemokine receptor has an α-bulge between positions 418 and 419; and **Right**: M2 muscarinic acetylcholine receptor (red; PDBid = 3uon [49]) superposed on the dopamine D3 receptor (cyan; PDBid = 3pbl [52]) as a reference. The M2 muscarinic receptor has an α-bulge between positions 428 and 429.

**Figure 13.** (**A**) Eleven adenosine 2A structures superposed. Light blue: 3vg9 [21] and 3vga [21] that each bind an inverse agonist; brown: 3eml [46], 3pwh [17], 3rey [17], 3rfm [17], 3uza [54] and 3uzc [54] that each bind an antagonist; red: 2ydo [14], 2ydv [14] and 3qak [55] that each bind an agonist. At some locations these three groups show systematic behavior that is illustrated in the blow-up of three representative structures (3vga, 3eml and 2ydo) in the panels **B**–**E**; (**B**) Helix II shows a systematic displacement of the area around the α-bulge towards helix III in the activated receptors; (**C**) Helix V in the activated receptors shows a systematic displacement of the area around the α-bulge towards helices III and IV; (**D**) Relative to the inverse agonist bound structures (cyan), the cytosolic side of helix V moves outward when an agonist is bound and inward when an antagonist is bound; and (**E**) The loop between helix VII and helix VIII behaves systematically (albeit in a hard to describe way) as function of the type of ligand bound, in line with the crucial role in the activation process for mobility of Tyr733.

**Figure 14.** Local superposition results of A2A adenosine receptor transmembrane helices. In this figure, helices are taken out of the structure and superposed without using the rest of the molecule. (**A**) Helix III becomes more regular upon activation. The side chain of one of Val-322 (known in many GPCRs to be crucial for binding the endogenous ligand) is indicated as a point of reference; (**B**) Helix IV is highly irregular at the cytosolic side. It is not clear if this is caused by the bound ligand or if it is caused by a crystal packing artifact; (**C**) Helix V is seen winding up more tightly going from inverse agonist, via antagonist, to agonist bound structures; (**D**) Helix VI neither tilts nor kinks upon activation. Instead, the entire helix rotates. A minor tightening of the cytosolic end of the helix is observed in the agonist bound form; and (**E**) Helix VII forms a bulge on the intracellular side upon activation while rotating toward the centre of the seven-helix bundle. 3qak shows a different Cα trace, which correlates with the absence of a structural water near this difference.

The article "Alpha-Bulges in G Protein-Coupled Receptors" was published in 2014. Journal: Int J Mol Sci.

**Figure 15.** (**A**) Seven β2 adrenoceptor structures superposed. Light blue: 2rh1 [56], 3d4s [57], 3ny8 [12] and 3ny9 [12] that each bind an inverse agonist; orange: 3nya [12] that binds to an antagonist; red: 3p0g [15] and 3sn6 [12] that each bind an agonist in combination with a nanobody and a trimeric G protein respectively to the cytosolic side. At some locations, these three groups show a systematic behavior that is illustrated in Panels **B**–**E**, which show a blow-up of three representative structures (light blue: 3ny8 bound to an inverse agonist; orange: 3nya bound to an antagonist; red: 3sn6 bound to an agonist and a trimeric G protein on the cytosolic side); (**B**) In helix II we observe a systematic motion of the area around the a-bulge towards helix III in the activated receptor; (**C**) In helix V, we observe a systematic motion of the area around the α-bulge towards helix III and helix IV in the activated receptor; (**D**) Relative to the inverse agonist bound structure (cyan) and the antagonist bound structure (orange), the cytosolic side of helix V moves outward when an agonist and a G-protein are bound as does helix VI; and (**E**) The loop between helix VII and helix VIII behaves systematically (albeit in a hard to describe way) as function of the type of ligand bound.

**Table 1.** Occurrence of α-bulges in the seven helices in the 84 GPCRs. Most α-bulges occur in helix II and helix V (near the ligand-binding pocket). The lipid receptors contain no α-bulges. α-Bulges were determined with DSSP 2.0. Helix VII generally contains a stretch of 3/10 helix near sequence position 720–725 (see Figure 9. The numbers 0, 1, and 2 indicate that we observed zero, one, or two bulges in that helix, respectively. In a few cases one extra turn of 3/10 helix is observed near the cytosolic end of Helix VII; these are indicated with −1.

Species	ID	TM1	TM2	TM3	TM4	TM5	TM6	TM7
Rhodopsin	1f88, 1gzm, 1hzx, 1l9h, 1u19, 2g87, 2hzy, 2i35, 2i36, 2i37, 2j4y, 2ped, 3c9l, 3c9m, 3oax	0	1	0	0	1	0	0
Opsin	2x72, 3cap, 3dqb, 3pqr, 3pxo, 4a4m	0	1	0	0	1	0	1
Rhod squid	2z73, 2ziy, 3aym, 3ayn	0	2	0	0	1	0	0
β1 AR	2vt4, 2y00, 2y01, 2y02, 2y03, 2y04, 2ycw, 2ycx, 2ycy, 2ycz, 4ami, 4amj, 4gpo	0	1	0	0	1	0	−1
β2 AR inact	2rh1, 3d4s, 3ny8, 3ny9, 3nya	0	1	0	0	1	0	−1
β2 AR act	3p0g, 3pds, 3sn6, 4lde, 4ldl, 4ldo	0	1	0	0	1	0	0
A2A inact	3eml, 3pwh, 3rey, 3rfm, 3uza, 3uac, 3vg9, 3vga, 4eiy	0	1	0	0	2 *	0	0
A2A act	2ydo, 2ydv, 3qak	0	1	0	0	2 *	0	1
CXCR4	3odu, 3oe0, 3oe6, 3oe8, 3oe9	0	0	0	1	1	0	0
Opioid	4djh, 4dkl, 4ea3, 4ej4	0	0	0	0	1	0	0
Lipid	3v2w, 3v2y	0	0	0	0	0	0	0
Serotonin 1B	4iaq, 4iar	0	1	0	0	1	0	0
Serotonin 2B	4ib4	1	1	0	0	1	0	0
CCR5	4mbs	0	0	0	0	1	0	0
PAR1	3vw7	0	0	0	0	1	1	0
NTSR1	4grv	0	1	0	0	1	0	0
Muscarinic	3uon, 4daj	0	1	0	1	1	0	0
Histamine H1	3rze	0	1	0	0	1	0	0
Dopamine D3	3pbl	0	1	0	0	1	0	0

* Bulge in Helix V of the A2A receptors is twice as long as in other receptors.

The article "Alpha-Bulges in G Protein-Coupled Receptors" was published in 2014. Journal: Int J Mol Sci.

## References

[1] PubMed http://www.ncbi.nlm.nih.gov/pubmed.

[2] Palczewski K., Kumasaka T., Hori T., Behnke C.A., Motoshima H., Fox B.A., le Trong I., Teller D.C., Okada T., Stenkamp R.E. (2000). Crystal structure of rhodopsin: A G protein-coupled receptor. Science.

[3] GPCR Network http://gpcr.scripps.edu/.

[4] Kouranov A., Xie L., de la Cruz J., Chen L., Westbrook J., Bourne P.E., Berman H.M. (2006). The RCSB PDB information portal for structural genomics. Nucleic Acids Res.

[5] Vroling B., Sanders M., Baakman C., Borrmann A., Verhoeven S., Klomp J., Oliveira L., de Vlieg J., Vriend G. (2011). GPCRDB: Information system for G protein-coupled receptors. Nucleic Acids Res.

[6] Horn F., Bettler E., Oliveira L., Campagne F., Cohen F.E., Vriend G. (2003). GPCRDB information system for G protein-coupled receptors. Nucleic Acids Res.

[7] Van Durme J., Horn F., Costagliola S., Vriend G., Vassart G. (2006). GRIS: Glycoprotein-hormone receptor information system. Mol. Endocrinol.

[8] Oliveira L., Paiva A.C., Vriend G. (1999). A low resolution model for the interaction of G proteins with G protein-coupled receptors. Protein Eng.

[9] Oliveira L., Hulsen T., Lutje Hulsik D., Paiva A.C., Vriend G. (2004). Heavier-than-air flying machines are impossible. FEBS Lett.

[10] Oliveira L., Paiva A.C., Sander C., Vriend G. (1994). A common step for signal transduction in G protein-coupled receptors. Trends Pharmacol. Sci.

[11] Rasmussen S.G., DeVree B.T., Zou Y., Kruse A.C., Chung K.Y., Kobilka T.S., Thian F.S., Chae P.S., Pardon E., Calinski D. (2011). Crystal structure of the β2 adrenergic receptor-Gs protein complex. Nature.

[12] Wacker D., Fenalti G., Brown M.A., Katritch V., Abagyan R., Cherezov V., Stevens R.C. (2010). Conserved binding mode of human β2 adrenergic receptor inverse agonists and antagonist revealed by X-ray crystallography. J. Am. Chem. Soc.

[13] Chun E., Thompson A.A., Liu W., Roth C.B., Griffith M.T., Katritch V., Kunken J., Xu F., Cherezov V., Hanson M.A. (2012). Fusion partner toolchest for the stabilization and crystallization of G protein-coupled receptors. Structure.

[14] Lebon G., Warne T., Edwards P.C., Bennett K., Langmead C.J., Leslie A.G., Tate C.G. (2011). Agonist-bound adenosine A2A receptor structures reveal common features of GPCR activation. Nature.

The article "Alpha-Bulges in G Protein-Coupled Receptors" was published in 2014. Journal: Int J Mol Sci.

[15] Rasmussen S.G., Choi H.J., Fung J.J., Pardon E., Casarosa P., Chae P.S., Devree B.T., Rosenbaum D.M., Thian F.S., Kobilka T.S. (2011). Structure of a nanobody-stabilized active state of the β2 adrenoceptor. Nature.

[16] Warne T., Serrano-Vega M.J., Baker J.G., Moukhametzianov R., Edwards P.C., Henderson R., Leslie A.G., Tate C.G., Schertler G.F. (2008). Structure of a β1-adrenergic G protein-coupled receptor. Nature.

[17] Doré A.S., Robertson N., Errey J.C., Ng I., Hollenstein K., Tehan B., Hurrell E., Bennett K., Congreve M., Magnani F. (2011). Structure of the adenosine A2A receptor in complex with ZM241385 and the xanthines XAC and caffeine. Structure.

[18] GPCR Activation: What Moves Where?. Van der Kant RWA.

[19] White J.F., Noinaj N., Shibata Y., Love J., Kloss B., Xu F., Gvozdenovic-Jeremic J., Shah P., Shiloach J., Tate C.G. (2012). Structure of the agonist-bound neurotensin receptor. Nature.

[20] Mason J.S., Bortolato A., Congreve M., Marshall F.H. (2012). New insights from structural biology into the druggability of G protein-coupled receptors. Trends Pharmacol. Sci.

[21] Hino T., Arakawa T., Iwanari H., Yurugi-Kobayashi T., Ikeda-Suno C., Nakada-Nakura Y., Kusano-Arai O., Weyand S., Shimamura T., Nomura N. (2012). G protein-coupled receptor inactivation by an allosteric inverse-agonist antibody. Nature.

[22] Katritch V., Reynolds K.A., Cherezov V., Hanson M.A., Roth C.B., Yeager M., Abagyan R. (2009). Analysis of full and partial agonists binding to β2-adrenergic receptor suggests a role of transmembrane helix V in agonist-specific conformational changes. J. Mol. Recognit.

[23] Rasmussen S.G., Choi H.J., Rosenbaum D.M., Kobilka T.S., Thian F.S., Edwards P.C., Burghammer M., Ratnala V.R., Sanishvili R., Fischetti R.F. (2007). Crystal structure of the human β2 adrenergic G protein-coupled receptor. Nature.

[24] Rey J., Deville J., Chabbert M. (2010). Structural determinants stabilizing helical distortions related to proline. J. Struct. Biol.

[25] Van Arnam E.B., Lester H.A., Dougherty D.A. (2011). Dissecting the functions of conserved prolines within transmembrane helices of the D2 dopamine receptor. ACS Chem. Biol.

[26] Cartailler J.P., Luecke H. (2004). Structural and functional characterization of pi bulges and other short intrahelical deformations. Structure.

[27] Worth C.L., Kreuchwig A., Kleinau G., Krause G. (2011). GPCR-SSFE: A comprehensive database of G protein-coupled receptor template predictions and homology models. BMC Bioinform.

[28] Deupi X. (2012). Quantification of structural distortions in the transmembrane helices of GPCRs. Methods Mol. Biol.

[29] Devillé J., Rey J., Chabbert M. (2009). An indel in transmembrane helix 2 helps to Trace the molecular evolution of class A G protein-coupled receptors. J. Mol. Evol.

The article "Alpha-Bulges in G Protein-Coupled Receptors" was published in 2014. Journal: Int J Mol Sci.

[30] Gonzalez A., Cordomí A., Caltabiano G., Pardo L. (2012). Impact of helix irregularities on sequence alignment and homology modeling of G protein-coupled receptors. Chembiochem.

[31] Isberg V., Vroling B., van der Kant R., Li K., Vriend G., Gloriam D. (2014). GPCRDB: An information system for G protein-coupled receptors. Nucleic Acids Res.

[32] Strobl C., Boulesteix A.L., Kneib T., Augustin T., Zeileis A. (2008). Conditional variable importance for random forests. BMC Bioinform.

[33] Toloşi L., Lengauer T. (2011). Classification with correlated features: Unreliability of feature ranking and solutions. Bioinformatics.

[34] Hofmann K.P., Scheerer P., Hildebrand P.W., Choe H.W., Park J.H., Heck M., Ernst O.P. (2009). A G protein-coupled receptor at work: The rhodopsin model. Trends Biochem. Sci.

[35] Vogel R., Sakmar T.P., Sheves M., Siebert F. (2007). Coupling of protonation switches during rhodopsin activation. Photochem. Photobiol.

[36] Fritze O., Filipek S., Kuksa V., Palczewski K., Hofmann K.P., Ernst O.P. (2003). Role of the conserved NPxxY(x)_5,6_F motif in the rhodopsin ground state and during activation. Proc. Natl. Acad. Sci. USA.

[37] Yohannan S., Faham S., Yang D., Whitelegge J.P., Bowie J.U. (2004). The evolution of transmembrane helix kinks and the structural diversity of G protein-coupled receptors. Proc. Natl. Acad. Sci. USA.

[38] Ceruso M.A., Weinstein H. (2002). Structural mimicry of proline kinks: Tertiary packing interactions support local structural distortions. J. Mol. Biol.

[39] Riek R.P., Rigoutsos I., Novotny J., Graham R.M. (2001). Non-α-helical elements modulate polytopic membrane protein architecture. J. Mol. Biol.

[40] Hong S., Ryu K.S., Oh M.S., Ji I., Ji T.H. (1997). Roles of transmembrane prolines and proline-induced kinks of the lutropin/choriogonadotropin receptor. J. Biol. Chem.

[41] Geetha V. (1996). Distortions in protein helices. Int. J. Biol. Macromol.

[42] Von Heijne G. (1991). Proline kinks in transmembrane α-helices. J. Mol. Biol.

[43] Conner A.C., Hay D.L., Simms J., Howitt S.G., Schindler M., Smith D.M., Wheatley M., Poyner D.R. (2005). A key role for transmembrane prolines in calcitonin receptor-like receptor agonist binding and signalling: Implications for family B G protein-coupled receptors. Mol. Pharmacol.

[44] Krieger E., Vriend G. (2002). Models@Home: Distributed computing in bioinformatics using a screensaver based approach. Bioinformatics.

[45] Hanson M.A., Roth C.B., Jo E., Griffith M.T., Scott F.L., Reinhart G., Desale H., Clemons B., Cahalan S.M., Schuerer S.C. (2012). Crystal structure of a lipid G protein-coupled receptor. Science.

The article "Alpha-Bulges in G Protein-Coupled Receptors" was published in 2014. Journal: Int J Mol Sci.

[46] Jaakola V.P., Griffith M.T., Hanson M.A., Cherezov V., Chien E.Y., Lane J.R., Ijzerman A.P., Stevens R.C. (2008). The 2.6 Ångstrom crystal structure of a human A2A adenosine receptor bound to an antagonist. Science.

[47] Murakami M., Kouyama T. (2008). Crystal structure of squid rhodopsin. Nature.

[48] Wu B., Chien E.Y., Mol C.D., Fenalti G., Liu W., Katritch V., Abagyan R., Brooun A., Wells P., Bi F.C. (2010). Structures of the CXCR4 chemokine GPCR with small-molecule and cyclic peptide antagonists. Science.

[49] Haga K., Kruse A.C., Asada H., Yurugi-Kobayashi T., Shiroishi M., Zhang C., Weis W.I., Okada T., Kobilka B.K., Haga T. (2012). Structure of the human M2 muscarinic acetylcholine receptor bound to an antagonist. Nature.

[50] Park J.H., Scheerer P., Hofmann K.P., Choe H.W., Ernst O.P. (2008). Crystal structure of the ligand-free G protein-coupled receptor opsin. Nature.

[51] Granier S., Manglik A., Kruse A.C., Kobilka T.S., Thian F.S., Weis W.I., Kobilka B.K. (2012). Structure of the δ-opioid receptor bound to naltrindole. Nature.

[52] Chien E.Y., Liu W., Zhao Q., Katritch V., Han G.W., Hanson M.A., Shi L., Newman A.H., Javitch J.A., Cherezov V. (2010). Structure of the human dopamine D3 receptor in complex with a D2/D3 selective antagonist. Science.

[53] Schwartz T.W., Frimurer T.M., Holst B., Rosenkilde M.M., Elling C.E. (2006). Molecular mechanism of 7TM receptor activation—A global toggle switch model. Annu. Rev. Pharmacol. Toxicol.

[54] Congreve M., Andrews S.P., Doré A.S., Hollenstein K., Hurrell E., Langmead C.J., Mason J.S., Ng I.W., Tehan B., Zhukov A. (2012). Discovery of 1,2,4-triazine derivatives as adenosine A2A antagonists using structure based drug design. J. Med. Chem.

[55] Xu F., Wu H., Katritch V., Han G.W., Jacobson K.A., Gao Z.G., Cherezov V., Stevens R.C. (2011). Structure of an agonist-bound human A2A adenosine receptor. Science.

[56] Cherezov V., Rosenbaum D.M., Hanson M.A., Rasmussen S.G., Thian F.S., Kobilka T.S., Choi H.J., Kuhn P., Weis W.I., Kobilka B.K. (2007). High-resolution crystal structure of an engineered human β2-adrenergic G protein-coupled receptor. Science.

[57] Hanson M.A., Cherezov V., Griffith M.T., Roth C.B., Jaakola V.P., Chien E.Y., Velasquez J., Kuhn P., Stevens R.C. (2008). A specific cholesterol binding site is established by the 2.8 Å structure of the human β2-adrenergic receptor. Structure.

[58] Berman H.M., Westbrook J., Feng Z., Gilliland G., Bhat T.N., Weissig H., Shindyalov I.N., Bourne P.E. (2000). The protein data bank. Nucleic Acids Res.

[59] Oliveira L., Paiva A.C.M., Vriend G. (1993). A common motif in G protein-coupled seven transmembrane helix receptors. J. Comput-Aided Mol. Des.

The article "Alpha-Bulges in G Protein-Coupled Receptors" was published in 2014. Journal: Int J Mol Sci.

[60] Vroling B., Thorne D., McDermott P., Attwood T.K., Vriend G., Pettifer S. (2011). Integrating GPCR-specific information with full text articles. BMC Bioinform.

[61] GPCRDB http://www.gpcr.org/7tm/.

[62] Konagurthu A.S., Whisstock J.C., Stuckey P.J., Lesk A.M. (2006). MUSTANG: A multiple structural alignment algorithm. Proteins Struct. Funct. Bioinform.

[63] Vriend G. (1990). WHAT IF A molecular modelling and drug design program. J. Mol. Graph.

[64] Vriend G., Sander C. (1991). Detection of common three-dimensional substructures in proteins. Proteins.

[65] Liaw A., Wiener M. (2002). Classification and regression by randomForest. R News.

[66] R Development Core Team (2008). R: A Language and Environment for Statistical Computing.

[67] Kabsch W., Sander C. (1983). Dictionary of protein secondary structure: Pattern recognition of hydrogen-bonded and geometrical features. Biopolymers.

[68] Joosten R.P., te Beek T.A., Krieger E., Hekkelman M.L., Hooft R.W., Schneider R., Sander C., Vriend G. (2011). A series of PDB related databases for everyday needs. Nucleic Acids Res.

[69] CMBI Protein Structure Bioinformatics Facilities.

[70] Index of Software DSSP.

